The article "The Sequential Influence of Creative Leadership and Organizational Environment on Strategic Performance" was retracted in 2023. Reasons: signs of a paper mill; suspected computer-generated content; unreliable results or conclusions; concerns about the data.

# The Sequential Influence of Creative Leadership and Organizational Environment on Strategic Performance

**DOI:** 10.1155/2022/5948806

**Published:** 2022-09-15

**Authors:** Dilshad Ahmed Salman, Khairi Ali Auso

**Affiliations:** Department of Business Administration, Near East University, Nicosia 99138, North Cyprus, via Mersin 10, Turkey

## Abstract

As a distinct form of leadership, the phenomena of creative leadership draw interest. Such leadership is crucial for developing and sustaining the operations of contemporary organizations and businesses. When it comes to boosting strategic effectiveness, the traits of creative leadership are crucial. This is a recognition of the paradoxes and contradictions present in life and a constructive evaluation of the team's creative potential. According to this study, a creative leader may greatly impact how effectively a strategy is implemented. This study explores the connection between innovative leadership and improved strategic performance. Developing nations' societies tend to undervalue innovative leadership's value in managing administration and enterprises. Unfortunately, it received little attention from academic sources and studies. Because of this, the primary goals of this study are to comprehend the ideas of creative leadership, the uniqueness of a leader's job as a manager, and the influence of creative leadership on strategic effectiveness. The goal of quantitative research is to comprehend how creative leadership may improve strategic effectiveness. Therefore, four hypotheses were tested in this study to show how creative leadership and strategic effectiveness are related. The research demonstrates how inventive leaders can enhance customer satisfaction through creative ideas. In conclusion, the strategic performance of a corporation depends on originality and creative leadership.

## 1. Introduction

First, it should be noted that successful firms and organizations typically have higher levels of dynamism and efficiency than other enterprises, underscoring the significance of leadership in today's management and company. Because of this, good leadership is necessary for leadership in the current day [1]. A manager and a leader have certain distinctions in every business or enterprise. The leader relies heavily on this position to build relationships with subordinates and can also be used to establish dominance. On the other hand, leadership is a unique form of management that places a greater emphasis on social relationships and interactions. Leadership involves greater contact between the participants since it is a more complex process [2].

The idea of creative leadership has been the focus of research in several nations since the turn of the twentieth century. “Creative leadership” is a style of leadership that is focused on working together to develop original solutions. People who lead intellectually do it by creating an environment that encourages it. Creative leadership is defined as taking the initiative, creating and resolving nonstandard tasks, being open to certain adjustments with others, and taking ownership of others' wellbeing. As a leader, users may generate new ideas that correspond with best practices in your sector by leveraging creativity. A creative outlook could also help users get ready for upcoming developments in their profession. The current society's economic and social developments have increased interest in innovative leadership. Innovation is very important to society's growth because it helps to find solutions to issues like these and strengthens the society's ability to respond. It is in charge of using new technology, typically, to efficiently and sustainably resolve problems in society. This is not by chance since a leader's innovative approach to solving challenges will be crucial to the future success of any business or organization, winning the competition, and the happiness of the workforce. The Davos Economic Forum listed 10 essential talents for 2020 in 2015 [3].

Evidently, among the required talents, creativity has come in third place. However, in today's world of fast change, traditional leadership is not always sufficient. A new unique quality is needed from the leader in order to increase strategic efficiency, create long-term strategic plans, and resolve unforeseen issues [4]. One of the key components of creative leadership is the quick evaluation of the issue's core and the creation of novel solutions. Otherwise, the odds of winning the competition are significantly diminished in a world of fast change.

Leadership is the effective deployment of several public resources to inspire others to take action in pursuit of common objectives. The first requirement for leadership in any size group, organization, or business is the availability of public resources [5]. We need to keep in mind that the leader's authority is explicitly recognized by law. In any situation, the team and society support the leader socially, psychologically, and emotionally. He will be able to guide them there. Despite the necessity of creative leadership in managing administration and enterprises, cultures in developing countries tend to undervalue it. Unfortunately, it took a poor position in scholarly publications and studies.

The “traditional concept of leadership” states that personal indicators are the foundation for leadership skills. A traditional leadership approach involves giving the leader based on power on existing customs. Examples from today include kings, theocrats, and a large number of business CEOs. The impact of those who came before almost all of the previous leaders was viewed as being conventional. This idea suggests that these indications might be inherited or acquired later in life. In the future, Frank Fiedler created the “situational concept of leadership”. Situational leadership is adjusting the management approach to accommodate the demands of the team or individual team members in each special circumstance or objective. There is not a leadership style that “fits everyone,” in their opinion [6]. Following this view, a person must establish an environment where he may self-actualize before presenting himself as a leader. It should be highlighted that in addition to skill, developing one's professional and personal traits is important to becoming a leader. Leadership abilities might fail if they are not cultivated over time. The fundamental characteristics of good leaders are the capacity to perceive and comprehend a situation in its whole, effectively communicate with others, earn others' trust, and make swift, informed judgments [7]. Any organization or society's dominant individual is its leader. A leader must have these characteristics in order to do this.

The contribution of the paper is as follows:

Enhancing strategic effectiveness is becoming more closely associated with innovative leadership. In addition, strategic efficiency, which primarily serves to increase a company's worth, is a measure of a business's long-term viability, especially for economic entities. All of these are seen as requirements for creative leadership. Consequently, a “manager-successor” connection is substituted for the traditional “manager-subordinate” one. Understanding the notions of creative leadership, the uniqueness of a leader's work as a manager, and how creative leadership impacts strategic success are thus the key goals of this study.

The paper is structured as follows: Section 1 indicates the introduction of the study.  Section 2 discusses about creative leadership and its role in a mobilizing a company. Methodology of the study is indicated in Section 3.  Section 4 indicates the result. Discussion about the study is indicated in Section 5; finally, Section 6 describes the conclusion of the study.

## 2. Creative Leadership and Its Role in Mobilizing a Company

The capacity to rally a group of people around a shared cause is the key characteristic of leadership. These characteristics, in particular, are becoming more crucial due to the growing significance of interpersonal relationships and the human dimension in management. Organizational change is based on the human dimension; as a result, individual change must be successful in order for organizational change to be really successful. Trindent understands the importance of the person in bringing about long-lasting change. In order to improve resource management by considering human causes, repercussions, and responses to coastal environmental problems, human aspects research integrates social science, humanities, and other subjects with natural science. Nearly every managerial task is seen as leadership at the same time. Leadership aspects are planning, constructing a management system, motivating, regulating, and controlling. However, the mechanisms that guarantee the reciprocal implementation of these duties are the main focus of leadership. These procedures include implementing managerial and communication choices and technology for people management [8].

The world is changing so quickly that new demands are being placed on leadership. It follows that since the old paradigm of connections in business and management is no longer functional, innovative individuals now have new options. The main characteristics of creative leadership include managing and going beyond efficiency. The objectives, words, presence, and actions of creative leaders are consistent, transparent, and honest. They establish an organizational culture that supports and encourages other people's ideas, gets rid of impediments, and sets up incentives to encourage the desired change. Every business and leader deals with a variety of issues daily. People frequently encounter these issues under the challenging socioeconomic conditions of our time, regardless of their line of work. Three key indicators of socioeconomic conditions are education, income, and population. The main methods for assessing socioeconomic status (SES) include looking at factors like occupation, income, and education. The way the global economy is structured is also drastically altering. A company's main concern is bringing in new customers and clients. We are now moving towards the era of inspiring people, as opposed to the information age. As a result, there is an increasing need for innovative leaders [9].

Torrance, the father of contemporary creativity, thought it was hard to fully characterize the phenomena of creativity in the middle of the twentieth century [10]. However, another indication of the intricacy of creativity is how difficult it is to define it accurately. As a result, it would be appropriate to discuss creativity and creative leadership in a particular setting. Employees with fewer than five years of experience were more likely to evaluate empowerment and performance favorably, according to the findings. In light of this finding, the authors of [11] recommend that Safeway Company raise and improve its performance by encouraging employees to offer the business feedback that enhances the services offered to clients.

Investing in the future leadership talent of a new generation is another aspect of creative leadership. Future leaders must be capable of cooperative collaboration in all areas of their work [8]. Creative leadership is, first of all, changing the existing mechanisms of influence on others. Creative leaders understand the necessity to influence others by developing their talents and practices. Meanwhile, they also try to create favorable conditions for the development of the creative abilities of subordinates. It is intended to achieve this through removing barriers to collaboration, learning from one another, and fostering creative collaboration. It is irrelevant in creative leadership whether the leader has a formal administrative position [12, 13]. However, his innovation will always come about due to collaboration, communication, and conflict resolution. This further suggests that those in leadership roles have the power to either foster or stifle team creativity.

The way creativity is seen as “service leadership” is another sign of creativity. A leader's primary responsibility is to bring his team's ideas and to think styles together [14]. Such leadership enhances each person's skills and helps him realize his potential for motivation. The ability of an organization to motivate its workforce is essential to its success. It refers to the level of commitment, enthusiasm, and intensity that a company's personnel bring to their daily job. Without it, organizations experience reduced levels of output, less productivity, and a greater risk of missing important goals. In order to achieve the goals of the organization, a leader must specifically motivate their team members to maximize their contributions. The performance of the organization and employee happiness are largely influenced by leadership and motivation. In this context, “selfless leadership” is also used to describe creative leadership. “Selfless leadership” is the ethical act of guiding people toward the achievement of set objectives and the greater good, representing the needs of others before one's own. A selfless leader should respect us, treat us with dignity, listen to us, understand us, give us credit, and educate us selflessly, show us the proper path to take, and never hesitate to point out our mistakes. They should guide us on the right way, encourage us to take the initial step, and nourish us for the future [9]. The leader should not attempt to keep things as they are in this situation.

On the contrary, he strives to develop new organizational opportunities while being open to innovation in a cultural and economic context that is quickly changing. Considering everything, we can conclude that the primary qualities of a creative leader are their capacity for productive work, their understanding of how emotions affect people, and their ability to anticipate the thoughts and intents of others. These characteristics are essential and fundamental for a creative leader. Additionally, there is a fundamental distinction between creative and conventional leaders. A creative leader has the ability to liberate the creativity in others. This kind of leadership focuses more than other types on developing an organizational culture that encourages and promotes creative thinking and problem-solving. The conventional leadership encourages cost-cutting, cost-saving, simplifying, and standardization. Managers that can demonstrate direction with their entire hand and are goal-oriented, and oriented results are important. A conventional leader, unlike a creative leader, is constantly concerned with maintaining the situation's stability and under his control. Creative leaders are typically not frightened of change because of their inventiveness, fast and flexible thinking, and innovation.

On the contrary, they can guide their teams toward similar objectives under challenging circumstances. Additionally, they are more adaptable to new circumstances than classical (conventional) leaders. It is a crucial quality of imaginative leaders. As we have already said, unlike a creative leader, a leader is constantly concerned with maintaining the status quo. Because of their inventiveness, fast and flexible thinking, and innovation, creative leaders are not frightened of change. Instead, they vary from the traditional leader because they are highly adaptable [15].

The necessity for specific abilities to operate in a changing environment due to the rapid expansion of global markets and technology is one of the primary reasons for the emphasis on creative leadership in Western countries [16]. Modern leaders rely on their abilities and sentiments rather than preexisting rules and standards when making judgments or statements about occurrences. Innovative leaders are always coming up with new ideas, implementing them, and attempting to expand their creative potential in the workplace. Instead of relying on traditional situations, today's leaders must be able to use their special abilities to make rapid, adaptable judgments in a changing environment. As a result, these leaders cannot rely on the achievements of others. This viewpoint concludes that creative leadership is based on individual abilities and knowledge [17].

### 2.1. Strategic Efficiency

A company's preplanned response to environmental changes to attain the desired result is known as strategy. Different labour, entrepreneurial, social, scientific, and technological tactics exist. Three major questions are addressed by strategic management: What is the business's present state? What condition should it be in after a given amount of time? What methods may be used to get this outcome? To provide answers to these queries, analytical techniques have been created. The management system, structure, and potential of human resources should be carefully examined to achieve the desired result while analyzing material, technical, organizational, and technological resources.

Five fundamental functions—strategic planning, organizing the execution of strategies, coordinating work on the implementation of strategic issues, motivating human resources to achieve strategic goals, and monitoring the strategy's implementation—are ensured by effective strategic management [14].

Therefore, in this study, the management actions include (a) gathering, storing, processing, and transmitting information; (b) developing and adopting management choices; (c) transferring management tasks to a managed object, and (d) exercising control over how decisions are carried out. Thus, the crucial function of leadership in strategic management has been represented in the criteria above [18].

### 2.2. The Role of Creative Leadership in the Implementation of the Strategy

As noted in the previous section, managers' leadership abilities are among the most critical prerequisites for successful plan execution. One of the important measures of leadership is how motivated employees are to carry out the planned changes [19]. At the same time, a leader must be able to persuade staff members and alter the company culture. The most challenging and complex process phase is often regarded as implementing these indicators. The company's management is responsible for clearly identifying the direction the organization will develop. Thus, they hold a significant position in this situation. However, knowing about the changes is insufficient. In addition, management should make an effort to reduce disputes that develop during the implementation of the strategic adjustments. To improve organizational performance, strategies can be designed to implement intended change, such as team-building initiatives. Change is inevitable, but there are many approaches to dealing with it, some of which are beneficial and others not [20].

The managers engaged may carry out the plan in various methods, including acting decisively or actively, delegating power, showing a keen interest in every aspect, and taking risks. The majority of businesses that have succeeded in putting their ideas into practice have management that is dynamic and effective, according to experience. The strategic manager takes the initiative, handles administrative duties, trains staff, and distributes resources to accomplish the goal [14, 21]. It is common practice to employ the Paul Hersey and Kenneth Blanchard model of strategical efficiency. The Hersey–Blanchard model states that there is no best leadership style. The idea encourages leaders to focus less on workplace difficulties and more on the people they manage and their talents. Unlike other leadership models, the Hersey–Blanchard model dismisses the idea that organizations require a singular style to leadership. The model suggests an alternative leadership approach that may be modified to the particulars of each workplace. This concept's strategic effectiveness, coaching, support, engagement, and exchange dimensions identify four fundamental circumstances in leadership [22]. The key factors that are considered in Hersey and Blanchard's situational theory is relationship, task, level of authority, and level of maturity as shown in Table 1.

In carrying out the strategy, the leader assumes five managerial obligations, including (1) monitoring events development, foreseeing potential issues, and examining elements that can obstruct the plan's execution. (2) Increasing business relationships and motivating team members to carry out a successful plan. (3) Continuing the organization's adaptive processes, continually looking for new chances, coming up with new concepts, and striving to surpass rivals in the competitive environment. (4) Guiding the implementation of strict moral principles and working to elevate the company. (5) Making modifications to boost the company's overall effectiveness and implementation of the plan [23].

Efficiency from an economic perspective refers to the strategies created to reach the objectives through the best possible means. Franklin Fisher asserts that a company's cash flow size determines how economically efficient it is. On the other hand, strategic effectiveness gauges a business's long-term viability [24]. Specialists' discontent with the organization's effectiveness measurement methods is rising. As a result, many businesses have doubts about the effectiveness of their systems. Companies with big, complex structures must examine more indications than organizations with smaller structures. However, only the indications used to forecast the future, assess the past, and inspire personnel are adequate in small businesses.

For measuring the effectiveness of structural units and functional areas, current research has focused on four key indicators: market assessment of the organization's activities in the financial markets (additional economic value, added value of equity capital); financial and accounting indicators (volume of income, profitability, cash receipts); and nonfinancial indicators (customer satisfaction, customer loyalty, and product compliance with technical requirements). As a result, we can see that two categories of future indicators may be utilized to help define an organization's strategy [25].

The main objective of strategic effectiveness should be to maximize the organization's value in management decision making. Therefore, innovative leaders use a variety of strategies to raise the most crucial measures of the organization's worth. Increasing an organization's strategic efficacy is its main challenge as a creative leader. It is sometimes thought that the key elements for leaders' success in managing an organization are intelligence, authority, self-confidence, energy, and professional knowledge because there is a direct correlation between the growth and success of any organization and its leadership style and managerial traits. However, research somewhat contradicts this assertion [7]. Therefore, only 25–30% of success relies on personal attributes, making them a secondary success factor in leadership. Instead, the management leadership style is the primary element that guarantees the firm's success. Therefore, it is crucial to emphasize two key characteristics of creative leadership to ensure strategic effectiveness: (1) Production orientation and (2) human orientation [15].

So, to be a creative leader, a high-level psychologist who can interact with every employee is a prerequisite. Creative leaders also possess a unique capacity to perceive psychological nuance. They also require other leaders' charisma and influence. Additionally, imaginative leaders have a social influence on the group, establishing subordinate relationships based on more humane standards. It is no accident that business owner today favor managers with more creative leadership traits when choosing top managers. In this instance, the leader takes control of the team, showcases their creative talents, and delivers greater product marketing and sales to boost the organization's strategic effectiveness. Because of their initiatives, innovative executives are accelerating the company's market share growth [20].

One of the most important elements in establishing strategic success is team motivation. Creative leaders reward the team and include them in decision making, which is different from typical managers and leaders in the incentive area. In addition, regular team members feel accountable for putting choices into action. The organization's successes are typically regarded as the responsibility of creative leaders. They are therefore interested in developing vertical communications, or lines of communication that go “top to bottom” and “from the bottom up.” In this scenario, the group activities and teamwork that occur become key determinants of the organization's strategic effectiveness [12]. Managers that adopt the position of creative leaders have faith in their staff members and encourage them on a moral and financial level to help them reach their objectives. As a result, the team assumes ownership in carrying out the strategic strategy.

Identifying each employee's capabilities has become one of the main elements in raising the strategic effectiveness of the firm in current times. A model where a worker is a regular system component and may be easily fired if required is not included [5]. The human component nowadays determines how productive and lucrative a business is, demonstrating how it is only natural to replace authoritarian and conventional leaders with innovative leaders. Bill Gates states, “Microsoft faces insolvency if 20 workers quit the business.” Therefore, it should be remembered that producing remarkable outcomes with the aid of regular people is the foundation of a strategically effective company [23]. The need to foster innovative thinking and an individualized approach for every employee simultaneously highlights the significance of creative leaders.

These hypotheses are formed by this research based on the study's underpinning theory:

**Hypothesis 1 .**

**(H1)**. Customers' satisfaction and desires and diversification of services are positively associated with employees' encouragement by creative leaders to solve workflow problems.

**Hypothesis 2 .**

**(H2)**. Customers' satisfaction and desires, as well as paying attention to the customers' complaints, are positively associated with participating employees of an organization in decision making and choosing innovative alternatives by creative leaders.

**Hypothesis 3 .**

**(H3)**. Customers' satisfaction and desires are positively associated with participating employees of an organization in creative leaders' decision-making.

**Hypothesis 4 .**

**(H4)**. Customers' satisfaction and desires are negatively associated with leaders' taking responsibility for making decisions by employees.

## 3. Methodology

In order to conduct this study, a questionnaire that 108 students completed at the Duhok Polytechnic University in northern Iraq was used as a qualitative approach. Strategic effectiveness and innovative leadership have been put at the center of attention. Creativity is the pioneering step of recognizing that something is possibly feasible. But innovation is more than just thinking; it is the act of putting information into practice in the face of obstacles and resistance. Utilizing creativity and innovation to manage people and projects is a part of an innovative leadership style. Innovative leaders typically encourage productivity through innovative and nontraditional strategies, going against the trend of the process. Strategic effectiveness is the primary focus of the creative leadership job. Strategic effectiveness is a method of thinking and performing as an organization to ensuring that its vision, purpose, and goals are accomplished. Users must look at how an organization strategy connects company goals to the methods they want to attain them and the tools they intend to employ in order to determine its efficacy and efficiency. A strategy is successful if it utilizes the available resources, allots them in accordance with their plan, and produces the desired outcomes. Several sub-variables are grouped up into these two primary variables. For instance, these three topics are emphasized under the question “Creative Leadership,” which is symbolized by an “X” in the tables: “solving issues and innovatively making decisions,” “innovative communication,” and “innovative thinking and planning.” Innovation communication entails the distribution of goods, services, or methods that differ from those currently in operation. The communication of innovation requires consideration of messaging, media, target audiences, and communication objectives. Only “customer satisfaction” is chosen to be explored and associated with the subvariables of creative leadership in the other variable (strategic effectiveness), questions shown as “Y”s in the tables.

## 4. Results

Table 2 shows the correlation between the variables. Y1 makes a significant correlation with “X1, X2, and X4,” with “*r* = 0.394, *p* = 0.000; *r* = 0.277, *p* = .004; *r* = 0.262, *p* = 0.006”, respectively. Then, Y2 makes it with “X1, and X2”, with “*r* = 0.192, *p* = 0.046; *r* = 0.324, *p* = 0.001”, respectively. In the same way, Y3 makes a significant correlation with “X2, X3, and X4”, with “*r* = 0.211, *p* = 0.028; *r* = 0.282, *p* = 0.003; *r* = 0.219, *p* = 0.004”, respectively.

## 5. Discussions

Customer satisfaction versus solving problems and making decisions in an innovative way.

The results demonstrate significant correlations between the variables under research, which is the major goal of the article to investigate the relationship between strategic success and creative leadership in emerging nations, according to Table 1. An ordinary leader looks on the present and understands how to manage an organization's day-to-day requirements. A strategic leader, on the other hand, looks to the future to develop new business prospects, products, or services for a company in order to accomplish its objectives. Leaders must be innovative in order to handle the ever-changing challenges of an unknown future. Innovative and productive executives enable businesses to develop cutting-edge goods and services and promote success. However, innovation is crucial at all levels of employment. There are multiple strong connections between the key variables in this study, which examines the relationship between “customer happiness” (strategic effectiveness) and “solving issues and making decisions in an inventive way” (creative leadership). The relationships between the minor variables are explained in Table 3:

The study's findings in Table 4 demonstrate how creative leadership may increase customer satisfaction. According to Table 4, customer happiness results from innovative leaders encouraging staff, including them in decision making and listening to their alternative answers. The last hypothesis, which the results did not support, also serves as a warning sign for whether or not creative leaders' failure to encourage their staff to assume responsibility leads to unsatisfied clients. Therefore, creative leaders must consider how they might encourage their team members to be more receptive to client demands and wishes in every situation.

## 6. Conclusion

There is no longer any debate among experts on the beneficial effects of innovative management and creative leadership on strategic effectiveness. Increasing strategic effectiveness is closely correlated with creative leadership traits. Additionally, the economic success of any business, corporation, or organization depends on a creative strategy. As a result of the quickening pace of change in the modern world, new styles of leadership are developing. Replacing the previous traditional and authoritarian leadership with new and creative ones is drawing attention as a natural process. As a result, a creative strategy's significance is growing, particularly in strategic management. It is essential to adjust to the most recent developments, make new decisions quickly to maximize earnings, guarantee that the business retains its place in the market, and inspire the team. Innovative and creative leadership is crucial to a company's strategic performance. One of the most important elements in attaining strategic goals is the mode of action and the leadership style. Developing personal attributes, inventiveness, and teamwork skills is crucial for establishing strategic effectiveness.

## Figures and Tables

**Table 1:** Leadership styles according to Paul Hersey and Kenneth Blanchard.

Performer training	The degree of focus on the task	Staff orientation coefficient	Leadership style
Not ready and not willing.	Maximum	Maximum	Give instructions
Not ready but willing to learn.	Middle	Middle	Support
He is ready but does not want to work	Down	Down	Attract
He is ready and willing to work	Down	Down	Date of authority

**Table 2:** Correlation between ‘customer satisfaction' and ‘solving problems and making decisions innovatively'.

Correlations							
Creative leadership							
				Solving problems and making decisions in an innovative way			
				*X1*	*X2*	*X3*	*X4*
	Customer satisfaction	Y1	Pearson correlation	0.394^*∗∗*^	0.277^*∗∗*^	0.184	0.262^*∗∗*^
			Sig. (2-Tailed)	0.000	0.004	0.056	0.006
			N	108	108	108	108
		Y2	Pearson correlation	0.192^*∗*^	0.324^*∗∗*^	−0.040	0.058
			Sig. (2-Tailed)	0.046	0.001	0.681	0.554
			N	108	108	108	108
		**Y3**	Pearson correlation	0.113	0.211^*∗*^	.282^*∗∗*^	0.273^*∗∗*^
			Sig. (2-Tailed)	0.242	0.028	0.003	0.004
			N	108	108	108	108

^*∗*^. Correlation is significant at the 0.05 level (2-tailed).^*∗∗*^. Correlation is significant at the 0.01 level (2-tailed). X1: I encourage subordinates to solve workflow problems in an innovative way. X2: Work to provide opportunities for subordinates to participate in decision-making, contributing to work development. X3: I take responsibility for the results after making my subordinates' decisions. X4: Choose innovative alternatives to solve work problems presented by subordinates. Y1: I seek to provide various services desired by clients, whether students or other entities. Y2: Adopt the diversification of services in order to meet the growing needs of students and keep pace with the labor market. Y3: I pay great attention to the complaints of customers from students or all other parties, as they represent the feedback of our concerns towards them.

**Table 3:** Correlation between subvariables.

	Correlation	r and *p* value	Interpretation
A	Y1	*r* = 0.394, *p* = 0.000	The more creative leaders encourage subordinates in their organizations to solve workflow problems, the clients will be more satisfied because the organization's employees try better to provide what customers desire.
	X1		
B	Y1	*r* = 0.277, *p* = 0.004	The more creative leaders work to provide opportunities for subordinates to participate in decision-making, which contributes to the development of work, and the clients will be more satisfied because the organization's employees try better to provide what customers desire.
	X2		
C	Y1	*r* = 0.262, *p* = 0.006	When creative leaders choose innovative alternatives to solve work problems presented by subordinates, they seek to provide various services desired by clients and promote customer satisfaction.
	X4		
E	Y2	*r* = 0.192, *p* = 0.046	Encouraging subordinates to solve workflow problems adopts the diversification of services.
	X1		
F	Y2	*r* = 0.324, *p* = 0.001	Allowing subordinates in decision making adopts the diversification of services.
	X2		
G	Y3	*r* = 0.211, *p* = 0.028	When creative leaders work to provide opportunities for subordinates to participate in decision-making, they pay great attention to the complaints of customers.
	X2		
H	Y3	*r* = 0.282, *p* = 0.003	When creative leaders take responsibility for the results after making decisions that subordinates participate in, subordinates pay great attention to customers' complaints.
	X3		
I	Y3	*r* = 0.273, *p* = 0.004	When creative leaders choose innovative alternatives to solve work problems presented by subordinates, subordinates pay great attention to the complaints of customers.
	X4		

**Table 4:** Summary of results.

Hypothesis	Findings
Customers' satisfaction and desires and diversification of services are positively associated with employees' encouragement by creative leaders to solve workflow problems.	Supported
Customers' satisfaction and desires, as well as paying attention to the customers' complaints, are positively associated with participating employees of an organization in decision-making and choosing innovative alternatives by creative leaders.	Supported
Customers' satisfaction and desires are positively associated with participating employees of an organization in creative leaders' decision making.	Supported
Customers' satisfaction and desires are negatively associated with leaders' taking responsibility for making decisions by employees.	Not supported

## Data Availability

No data were used to support the study.
